# Effect of Self-Transcendence Theory Combined with Comprehensive Nursing Intervention under Tumor Nutrition Education on Symptom Improvement, Nutritional Status, and Positive Psychology of Elderly Patients with Gastric Cancer

**DOI:** 10.1155/2022/6084732

**Published:** 2022-07-12

**Authors:** Xijuan Cui, Tao Shan, Lina Qiao

**Affiliations:** Department of General Surgery, The First Affiliated Hospital of Xi'an Jiaotong University, Shanxi, Xi'an 710061, China

## Abstract

**Objective:**

To explore the value of self-transcendence theory combined with comprehensive nursing intervention under oncological nutritional education on improvement in symptoms, nutritional status, and positive psychology of elderly patients with gastric cancer (GC).

**Methods:**

A total of 98 elderly patients with GC in the First Affiliated Hospital of Xi'an Jiaotong University from January 2021 to December 2021 were enrolled. All these patients were arbitrarily assigned into the observation group (*n* = 49) and control group (*n* = 49). The controlled patients accepted the regular oncological nutritional education. The cases of the observation group were given comprehensive nursing care based on the self-transcendence theory and oncological nutrition education. The symptom remission rate, subjective global assessment (PG-SGA) score, self-transcendence scale score, incidence of malnutrition, Hamilton Anxiety (HAMA) scale score, Hamilton Depression (HAMD) scale score, and Newcastle satisfaction with nursing scale (NSNS) score were observed.

**Results:**

The remission rate of symptoms in the observation group was higher than that of the control group after the nursing care. Following nursing, the PG-SGA score of the observation group was lower than that of the control group (*p* < 0.05). The score of the self-transcendence scale in the observation group was higher than that of the control group after nursing (*p* < 0.05). The incidence of malnutrition in the observation group was significantly lower than that of the control group. After nursing, the scores of the HAMA scale and HAMD scale in the observation group were lower than that of the control group (*p* < 0.05). The NSNS score of the observation group was statistically higher than that of the control group following nursing.

**Conclusion:**

The application value of self-transcendence theory combined with comprehensive nursing care under oncological nutritional education is more significant in elderly patients with GC, which is more helpful to enhance symptoms and nutritional status and control the incidence of malnutrition. Thus, it is able to reduce anxiety and depression and the rate of adverse reactions related to surgery-assisted chemotherapy as well.

## 1. Introduction

Gastric cancer (GC) is one of the commonest malignant tumors and the global incidence is trending upwards [1]. According to the statistics of the International Agency for Research on Cancer in 2018, the incidence of GC ranks fifth and the mortality rate ranks third among all malignant tumors. About 1 million new cases of GC are diagnosed each year, and approximately 783,000 of all cancer patients die from GC [1, 2]. More than 70% of all new cases of GC are from developing countries, about 50% from East Asia. Chinese cases account for 42.6% of global GC cases and 45.0% of global GC deaths, which is an important public health problem [2]. With the spread of early GC screening programs and continued advancements in GC therapies, the survival rates and survival times of GC patients have already continued to improve. However, the adverse effects of the antineoplastic therapy and physiological effects of cancer itself can cause negative emotions in oncology patients [3]. Studies have shown that psychological pain has a negative impact on antitumor therapies, reducing patients' quality of life, making patients less compliant with treatment, and even reducing long-term survival rates for tumor patients [4]. Therefore, the nutritional status, quality of life, and psychological pain of tumor patients have been paid more attention.

Previous studies have demonstrated that the nutritional status of oncology patients is closely related to inflammation, quality of life, and psychological distress [5]. Due to the systemic effects of metabolic changes and inflammatory reactions caused by tumors, the incidence of malnutrition is high. 40–80% of patients suffer from malnutrition and about 20% of tumor patients die of malnutrition [6]. In addition, malnutrition reduces the patient's tolerance to surgery and radiotherapy adjuvant chemotherapy, decreases the patient's quality of life, and affects the patient's clinical outcome [7]. Therefore, nutritional therapy for tumor patients have become an important part of multidisciplinary comprehensive antitumor therapy [8]. Self-transcendence means that in the face of life events, individuals can adjust their personal concepts and give full play to their potential, so as to learn to coexist with diseases or special events and reach a new level [9]. Self-transcendence is a domain theory in nursing, which was first put forward by Reed, professor at the School of Nursing of the University of Arizona in 1991 [10]. Reed believes that as older people age, their ability to perform everyday tasks will inevitably be affected, but that aging is a process of maturity of mind and life experience, not a process of deterioration [11]. There have been a few clinical studies combining self-transcendence theory with integrated care interventions under oncology nutrition education.

## 2. Patients and Methods

### 2.1. General Information

A total of 98 patients with GC hospitalized in the First Affiliated Hospital of Xi'an Jiaotong University from January 2021 to December 2021 were enrolled. All GC patients were arbitrarily assigned into the observation group (*n* = 49) and control group (*n* = 49). The controlled patients accepted the regular oncological nutritional education. The cases of the observation group were given comprehensive nursing care based on self-transcendence theory and oncological nutrition education. Inclusion criteria were as follows: the patients were older than 60 years who were diagnosed as GC by histopathology and received postoperative adjuvant chemotherapy, the participants without distant metastasis of organs, the participants without contraindication of surgery-assisted chemotherapy and it was estimated that 6 courses of surgery-assisted chemotherapy can be completed, the participants without infection or other autoimmune disorders (such as vasculitis and rheumatoid arthritis), and the patients who could voluntarily cooperate and complete nutritional assessment, nutritional treatment, dietary survey and quality of life assessment. Exclusion criteria were as follows: accurate information on dietary surveys, nutritional assessments, quality of life, psychological distress, and subjective well-being that cannot be obtained from patients or their families; patients with autoimmune diseases; patients with serious concomitant diseases (chronic heart, lung disease, severe liver, and kidney dysfunction.); and the patients who failed to complete nutritional treatment.

### 2.2. Treatment Methods

#### 2.2.1. Technical Route

The technical route is shown in Figure 1.

#### 2.2.2. Intervention Scheme

The control group was given the routine oncological nutritional education. The nutrition treatment team was composed of doctors, dietitians, and nurses. According to the general principles of nutritional treatment of tumor and following the five-step model of nutritional treatment, the individualized nutritional treatment plan was formulated and implemented [12]. When receiving nutritional treatment after operation for GC, the first stage was nutrition education plus diet, the second stage was oral nutrition supplement, the third stage was enteral nutrition, the fourth stage was partial parenteral nutrition + partial enteral nutrition, and the fifth stage was total parenteral nutrition [13]. The diet of the patients was formulated by the nutrition treatment group according to the patients' eating habits, eating conditions, gastrointestinal reactions, and consumption capacity and carried out nutrition education to the patients and their families combined with food models and food exchange portions to ensure the compliance of the patients and their families with the diet [14]. Meanwhile, the patient's personal nutrition treatment file was established to record the patient's nutrition treatment plan, implementation, compliance, and obstacles, requiring patients to monitor and adjust the nutrition treatment program to the nutrition department during each operation [15]. During this period, the patients could contact the dietitian through WeChat or telephone to communicate in a timely manner the problems that were displayed in the implementation of their diet or nutrition treatment.

The observation group was given a comprehensive nursing intervention based on self-transcendence theory and tumor nutrition education. (1) The formulation of nursing strategy: the keywords of “senile GC,” “self-transcendence,” “nursing,” and “nutrition education” were searched in some well-known databases such as Zhi.com, Wanfang, and VIP, and summed up the nursing strategies and design methods based on self-transcendence theory. Nursing strategies were formulated under the guidance of the self-transcendence theory nursing strategy, combined with the experience of experts in the field of psychology, senior nurses, and patients' own conditions in our hospital. (2) The implementation of nursing strategy: it can be assigned into four stages according to the connotation of self-transcendence theory. The first stage (caring for inner activities and promoting self-awareness): collective cognitive intervention 50 min was conducted in the first and second weeks to let patients communicate, internalize and understand each other, introduce emotion theory, explore patients' inner activities such as cognition, belief, will, and desire, enhance self-emotional management, and get out of the predicament. In the third week, we conducted group meditation practice 30 min, played meditation music in a loop, guided self-adjustment through meditation training, and improved self-acceptance. The fourth week of one-to-one intervention in 20 min let patients objectively show their own personality characteristics in the form of language and pictures, excavate, and deepen their self-understanding. The second stage (expanding self-boundaries and caring for others): in the fifth week, we conducted collective intervention, organized symposia among patients, encouraged the sharing of disease and treatment energy among patients, thought for others, constantly transcended their own thinking, and established a good relationship between patients. Care, encourage, help others, and take the initiative to express their feelings to relatives and friends; The third stage (reviewing the past, cherishing the present, and looking forward to the future): week 6, one-on-one intervention in 30 min allows patients to face up to the past, share their past life events, learn to relax, reshape, and adapt to diseases and other living conditions, make full use of external social support resources, strengthen and shape hope, and find the meaning of life. Cherish the present and look forward to the future with a positive attitude, feel the sense of trust, belonging, and cohesion, and achieve self-transcendence. The fourth stage (improving individual mental strength): collective intervention in 40 min at the 7th and 8th week was conducted to introduce the theoretical connotation of self-transcendence and guide patients how to transcend and accept themselves. Select quotations such as soul chicken soup to guide patients to think and discuss themselves, fully tap their inner self-regulation strength, and strengthen their spiritual strength.

### 2.3. Observation Index

The main observations indexes include the symptom improvement rate. The improved solid tumor evaluation standard (mRECIST) was adopted to evaluate. The complete remission indicated no enhancement of all lesions in the arterial enhancement phase. The partial remission meant the sum of the diameter of contrast-enhanced lesions in the arterial phase decreased by at least 30%. The disease progression was assessed though the sum of the diameter of contrast-enhanced lesions in the arterial phase increased by at least 20%. The disease stability was indicated neither partial remission nor disease progression. The clinical disease control rate = (complete remission + partial remission + disease stability) number of cases/total number of cases × 100%:

1. The subjective global assessment (PG-SGA) scores were observed. The PG-SGA is a nutrition assessment method specially designed for tumor patients, which is developed from subjective overall assessment [16]. It is composed of patient self-assessment part (4 aspects) and medical staff evaluation part (3 aspects). The scores of 7 aspects are added together to get a final score for qualitative evaluation. 0 or 1 score is considered as good nutritional status; the score from 2 to 8 is indicated as mild to moderate malnutrition. More than 9 points are seen as severe malnutrition.
2. Observe the self-transcendence scale scores. The self-transcendence scale compiled and processed by Reed was used to evaluate the self-transcendence ability, including 10 items, with a total score of 0–50 points. The higher the score is, the stronger the self-transcendence ability.
3. Observe the incidence of malnutrition.
4. Observe the scores of the Hamilton Anxiety (HAMA) scale and Hamilton Depression (HAMD) scale in the two groups. The HAMA scale score of <7 points indicated the patient has no anxiety [17]. A score of 7–13 points indicated the possibility that the patient has anxiety. A score from 14 to 20 indicated the patient must have anxiety. The 21–28 score indicated that the patient has obvious anxiety. A score of ≥29 indicated that the patient's anxiety is serious [18]. The HAMD scale score of <8 indicated that the patient is normal and has no depression [19]. A score between 8 and 20 points indicated that the patient has depression. A score between 8 and 20 points represents the patient must have depression. A score of more than 35 means that the patient has serious depression.
5. The scores of Newcastle satisfaction with nursing scale (NSNS) was observed. There are 19 test items in the NSNS scale [20]. Each item is evaluated with a score from 1 to 5, including 1 (very dissatisfied), 2 (dissatisfied), 3 (general satisfaction), 4 (satisfied), and 5 (very satisfied).

### 2.4. Statistical Analysis

The statistical analysis was performed by using the SPSS 24.0 software. The statistical graphics were drawn by GraphPad Prism 8.0. The measurement data in accordance with normal distribution were presented by mean ± standard deviation. The paired sample *t*-test was adopted for intragroup comparison and the independent sample *t*-test was adopted for intergroup comparison. The intragroup comparison was carried out by using the paired sample nonparametric test and intergroup comparison was carried out by using the independent sample nonparametric test. The grade data were examined by the Fisher accurate method. *P* less than 0.05 exhibited statistical significance.

## 3. Results

### 3.1. The Symptom Improvement Rate Was Observed

The remission rate of symptoms in the observation group was higher compared to the control group (*p* < 0.05, Table 1).

### 3.2. The Scores of PG-SGA Scales Were Observed

Before nursing, there exhibited no significant difference in the PG-SGA score (*p* > 0.05). After nursing, the PG-SGA score of the observation group was lower than that of the control group (*p* < 0.05, Table 2).

### 3.3. The Score of Self-Transcendence Scale

Before nursing, there exhibited no significant difference in the score of self-transcendence scale (*p* > 0.05). After nursing, the score of self-transcendence scale in the observation group was higher than that of the control group (*p* < 0.05, Table 3).

### 3.4. The Incidence of Malnutrition between the Two Groups

The incidence of malnutrition in the observation group was lower than that of the control group (*p* < 0.05, Table 4).

### 3.5. The Scores of HAMA Scale and HAMD Scale between Two Groups

Before nursing, there exhibited no significant difference in the HAMA scale score and HAMD scale score (*p* > 0.05). After nursing, the scores of HAMA scale and HAMD scale in the observation group were lower than that of the control group (*p* < 0.05), as given in Tables 5 and 6.

### 3.6. The NSNS Score between Two Groups

Before nursing, there exhibited no statistical difference in NSNS scores (*p* > 0.05). After nursing, the NSNS score of the observation group was higher than that of the control group (*p* < 0.05, Table 7).

## 4. Discussion

According to the statistics of the China National Cancer Center in 2018, among all malignant tumors, the incidence of GC is the second and the mortality rate is the third [21–23]. Global cancer survival monitoring data show that about 80% of GC patients in China are in advanced stage at the time of diagnosis, and the survival rate of 5 GC patients is 35.9% [24]. Because gastric surgery has the most complications and lasts the longest in all gastrointestinal operations, gastrointestinal resection or diversion and loss of gastric juice caused by surgery will cause a variety of nutritional digestion and absorption disorders. Therefore, malnutrition in patients with GC is frequent, severe, persistent, and complex and is one of the tumors with the most serious impact on nutritional status [25]. Meanwhile, the lack of knowledge of tumor nutritional treatment and the low rate of correct nutritional behavior, especially poor understanding of protein foods, blind taboo, increase the risk of malnutrition, malnutrition in tumor patients lead to surgery, radiotherapy, and chemotherapy complications, and chemotherapy toxicity increases and not only makes the tumor itself cannot get timely and effective treatment but also increases the treatment-related mortality, affecting the prognosis and survival rate of tumor patients, reduces the quality of life of tumor patients, prolongs the length of stay, and increases medical expenses [6]. Meanwhile, malnutrition also limits the choice of treatment options for tumor patients. In addition, almost all the elderly patients with GC experienced the process of doubt, denial, fear, sadness, despair, and helplessness in the process of diagnosis and treatment. Psychological pain affects tumor patients in dealing with tumors, reducing somatic symptoms, antitumor therapy, affecting treatment compliance, reducing patients' quality of life, and even reducing the long-term survival rate of tumor patients [7]. Therefore, for elderly patients with GC, how to take effective nursing measures for enhancing their nutritional status and psychological status are of great significance to promote the treatment effect and strengthen the quality of life of the patients.

The nutritional status of tumor patients is closely related to their prognosis. Nutritional therapy has become an important part of multidisciplinary comprehensive treatment of cancer, which should run through the whole process of antitumor therapy for patients with GC [26]. The purpose of nutritional therapy for patients with GC is to provide sufficient nutrients for the body, reduce metabolic disorders, enhance physiological and immune function, improve symptoms such as anorexia and fatigue, reduce or avoid side effects of antitumor therapy, reduce the risk of treatment interruption, help patients get through the treatment stage safely, and promote their quality of life. In addition, nutritional therapy can also increase the tolerance of tumor patients to surgery, radiotherapy, and chemotherapy, reduce surgical complications, reduce the interruption of radiotherapy and chemotherapy, and also reduce the adverse reactions of radiotherapy and chemotherapy. But, during the treatment, elderly patients with GC are under psychological and physical pressure, and they are easy to escape from reality and fall into helpless and negative situations. Self-transcendence theory originated from the field of physiology, through comprehensive psychological assessment, so that patients independently participate in the management of stress events in various dimensions [27]. Therefore, this research carried out a study to explore the value of comprehensive nursing intervention under self-transcendence theory combined with tumor nutrition education on symptom improvement, nutritional status, and positive psychology of elderly patients with GC.

Our results have suggested the remission rate of symptoms in the observation group was higher than that of the control group after the nursing care. Following nursing, the PG-SGA score of the observation group was obviously lower than that of the control group. The score of the self-transcendence scale in the observation group was higher than that of the control group after nursing. The incidence of malnutrition in the observation group was significantly lower than that of the control group. After nursing, the scores of the HAMA scale and HAMD scale in the observation group were lower than that of the control group. The NSNS score of the observation group was statistically higher than that of the control group following nursing. It is proved that the comprehensive nursing intervention based on the self-transcendence theory combined with tumor nutrition education has a more significant application value in elderly GC patients, which is more conducive to improving symptoms and nutritional status, controlling the incidence of malnutrition, reducing anxiety and depression, and reducing surgical assistance [28]. Chemotherapy-related adverse reaction rates: this is mainly because there is a positive correlation between the level of self-transcendence and mental health, and improving the level of self-transcendence is an effective means to restore and maintain mental health, and it is also the focus of nursing work [29]. Applying self-transcendence theory and tumor nutrition education to the clinical nursing work of elderly patients with GC can fully tap the power of personal inner self-regulation, establish connections with the internal and external environment, expand the personal upper limit, reshape and adapt to the disease and other living conditions, and make full use of the external environment [30]. Social support resources, strengthen and shape hope, seek meaning in life, make them aware of the dangers of malnutrition, actively cooperate with nutritional treatment, and enhance the psychological state of patients [31]. Thomas et al. found that when facing the major life event of cancer, female breast cancer patients will summarize their own life experience, reflect on the purpose and meaning of life, and finally overcome the disease and restore their mental health [32]. It is suggested that nurses should incorporate self-transcendence into the overall dimension of the patient's physical and mental functions, help patients summarize past experiences, rebuild future goals, and achieve self-transcendence through comprehensive reflection to improve their mental health [33]. Haugan explored the relationship between self-transcendence and mental health of nursing home patients, found that self-transcendence is a favorable factor to promote the mental health of patients, and pointed out that nurses should start from the internal and external dimensions of self-transcendence, encourage patients to reflect on themselves, and help others [34]. In addition, there was also a clear correlation between self-transcendence and depression levels. Yang Zhilan et al. found that the higher the level of self-transcendence in the elderly, the more positive life experiences and emotions they have, and a higher level of self-transcendence can improve the ability of the elderly to deal with life events, thereby reducing negative emotions and [35] reducing the incidence of depression. The results of Haugan et al. also confirmed the negative relationship between self-transcendence and depression and pointed out that actively connecting with the outside world and helping others can prevent or reduce depression [36]. Meanwhile, effective nurse-patient communication can promote patients' self-acceptance and self-adjustment, strengthen the patient's connection with the external environment, stimulate the patient's reflection, and have a positive impact on the patient's self-transcendence and mental health [35, 37].

Conclusively, the comprehensive nursing healthcare based on the combination of self-transcendence theory and regular oncological nutritional education has a more significant applied value in elderly patients with GC. It is able to facilitate enhanced nutritional status, control the incidence of malnutrition, reduce anxiety and depression, and reduce the adverse effects of surgical adjuvant chemotherapy.

## Figures and Tables

**Figure 1:** Technical route.

**Table 1:** The remission rate of symptoms in two groups.

Score	Complete remission (*n*/%)	Partial remission (case/%)	Disease progression (case/%)	Disease is stable (case/%)	Symptom improvement remission rate (case/%)
C group (*n* = 49)	20 (40.82)	9/18.37	8/16.33	12/24.48	29/59.19
O group (*n* = 49)	29/59.18	10/20.41	6/12.24	4/8.17	39/79.59
*χ* ^2^					4.804
*P*					0.028

**Table 2:** The score of PG-SGA scale in two groups.

PG-SGA scale score (points)	Before nursing	After nursing	*t* value	*P* value
C group (*n* = 49)	7.54 ± 1.19	3.72 ± 0.17	22.245	<0.05
O group (*n* = 49)	7.85 ± 1.12	2.19 ± 0.03	35.362	<0.05
*t*	1.328	62.041		
*P*	0.187	<0.05		

**Table 3:** The score of self-transcendence scale in two groups.

Self-transcendence scale score (points)	Before nursing	After nursing	*t* value	*P* value
C group (*n* = 49)	15.12 ± 1.39	18.19 ± 1.25	11.496	<0.05
O group (*n* = 49)	15.14 ± 1.44	29.23 ± 2.35	36.040	<0.05
*t*	0.069	29.033		
*P*	0.944	<0.05		

**Table 4:** The incidence of malnutrition between the two groups.

Group	Incidence of malnutrition (case/%)
C group (*n* = 49)	15/30.61
O group (*n* = 49)	5/10.20
*χ* ^2^	6.282
*P*	0.012

**Table 5:** The score of HAMA scale in two groups.

HAMA scale score (points)	Before nursing	After nursing	*t* value	*P* value
C group (*n* = 49)	19.29 ± 1.64	12.59 ± 0.32	28.068	<0.05
O group (*n* = 49)	19.31 ± 1.65	8.36 ± 1.14	38.219	<0.05
*t*	0.060	25.007		
*P*	0.952	<0.05		

**Table 6:** The score of HAMD scale in two groups.

HAMD scale score (points)	Before nursing	After nursing	*t* value	*P* value
C group (*n* = 49)	22.11 ± 1.25	14.02 ± 2.17	22.613	<0.05
O group (*n* = 49)	22.17 ± 1.39	9.58 ± 1.11	49.544	<0.05
*t*	0.225	12.751		
*P*	0.823	<0.05		

**Table 7:** The NSNS scores of the two groups.

NSNS scale score (points)	Before nursing	After nursing	*t* value	*P* value
C group (*n* = 49)	78.19 ± 3.77	81.77 ± 4.21	4.434	<0.05
O group (*n* = 49)	78.21 ± 3.79	89.88 ± 5.01	13.004	<0.05
*t*	0.026	8.675		
*P*	0.979	<0.05		

## Data Availability

The datasets used and analyzed during the current study are available from the corresponding author upon request.
